# An Unsupervised 3D Image Registration Network for Brain MRI Deformable Registration

**DOI:** 10.1155/2022/9246378

**Published:** 2022-10-03

**Authors:** Min Huang, Guanyu Ren, Shizheng Zhang, Qian Zheng, Huiyang Niu

**Affiliations:** Software College, Zhengzhou University of Light Industry, Zhengzhou 450000, China

## Abstract

In recent years, deep learning has made successful applications and remarkable achievements in the field of medical image registration, and the method of medical image registration based on deep learning has become the current research hotspot. However, the performance of convolutional neural networks may not be fully exploited due to neglect of spatial relationships between distant locations in the image and incomplete updates of network parameters. To avoid this phenomenon, MHNet, a multiscale hierarchical deformable registration network for 3D brain MR images, was proposed in this paper. This network was an unsupervised end-to-end convolutional neural network. After training, the dense displacement vector field can be predicted almost in real-time for the unseen input image pairs, which saves a lot of time compared with the traditional algorithms of independent iterative optimization for each pair of images. On the basis of the encoder-decoder structure, this network introduced the improved Inception module for multiscale feature extraction and expanding the receptive field and the hierarchical forecast structure to promote the update of the parameters of the middle layers, which achieved the best performance on the augmented public dataset compared with the existing four excellent registration methods.

## 1. Introduction

Medical image registration is the process of optimally aligning the moving image with the reference image through a certain spatial transformation, and it is the preliminary work for some medical image analysis operations such as identification and segmentation. The quality of registration directly affects the effect of its task and the follow-up task, so the research on medical image registration technology has far-reaching and realistic significance. Depending on the type of spatial transformation, image registration includes linear transformation and nonlinear transformation. The linear transformation includes rigid registration and affine registration. It is an overall transformation for the global image and is often used as a preregistration operation for complex multistage registration [1]. Deformation registration is nonlinear registration, which allows local elastic transformations of images, and can capture irregular deformations between tissues or organs to achieve fine alignment between images [2]. Researchers have proposed many traditional intensity-based or feature-based iterative algorithms for deformable medical image registration [3–5]. These algorithms use multiple iterations to continuously update and optimize the transformation parameters by calculating the similarity between the moving and the reference images. Although this kind of method has achieved remarkable results on many datasets, it is not suitable for clinical medical research that has strict requirements on computing time and efficiency due to its huge time consumption and the operational complexity caused by manual parameter adjustment. In recent years, deep learning, especially the convolution neural network (CNN), has had a subversive impact on the field of computational vision, including image classification, image segmentation, and target detection. The deep learning-based registration method replaces the iterative optimization process of the traditional algorithm by using a trained model to achieve fast registration of an unseen pair of image volumes. It has developed rapidly and has become the main direction of medical image registration research today by virtue of its excellent computing speed and accuracy. The registration methods based on deep learning were originally proposed in the form of supervised learning, but obtaining the ground truth required by supervised learning is not trivial, because the ground truth contains a large amount of annotation data. The ground-truth deformation field or region of interest (ROI) labels required for supervised training often need to be manually labeled by experts [6, 7], but the acquisition cost is expensive and highly dependent on professional knowledge. Therefore, there were methods to replace the manual annotation with random transformation synthesis [8] or the results obtained by traditional algorithms [9, 10], but these methods will restrict the upper limit of the registration accuracy.

The emergence of the spatial transformer network (STN) [11] has greatly promoted the development of unsupervised learning. STN, a differentiable module, can be directly embedded in the registration model, generate a sampling grid according to the deformation field predicted by the neural network, and warp the moving image through multilinear interpolation to obtain the deformed image, which makes it possible to calculate the image similarity in the training process. De Vos et al. [12] proposed the first unsupervised registration network based on image similarity, which takes the similarity between the deformed image and the reference image as the loss function, making end-to-end unsupervised network training possible. After that, De Vos et al. [13] first proposed an unsupervised affine and deformable image registration framework, which integrated linear and nonlinear registration in one architecture by stacking multiple CNNs, achieving a coarse-to-fine registration. Fan et al. [14] proposed BIRNet, which introduced the deformation field evaluated by the traditional registration algorithm as the ground truth on the basis of the unsupervised learning strategy to guide loss attenuation in a dual-supervised way. At the same time, the similarity loss is calculated by using the deformed image patches with different resolutions, so as to speed up the convergence of the network. These algorithms all have good registration performance, but they are all based on 3D image patches. This situation often causes the convolution neural network to ignore the long-range spatial relationship in the image, which restricts the network to predict relatively large local deformation. Balakrishnan et al. [15, 16] proposed the VoxelMorph framework to realize the registration of the entire image. The VoxelMorph framework defines the registration process as a function, parameterizes the function through the CNN network, and uses the complete 3D image as training data to continuously update and optimize the parameters. The trained network can achieve one-pass registration of unseen input images, which achieves unsupervised registration of full-size images. Zhao et al. [17] also designed an unsupervised deformation network Volume Tweening Network (VTN), which can solve large displacement deformation end-to-end by recursively cascading multiple deformable networks. However, due to the increase of CNN depth and downsampling times, to keep the output displacement vector field matching the input image, VTN has more stringent requirements on the size of the input image and device memory.

In this paper, we proposed a novel unsupervised fully convolutional neural network for 3D brain MR image registration, called multiscale hierarchical deformable registration network (MHNet). While abandoning the manual parameter tuning of traditional registration methods and the ground truth requirements of supervised learning networks, MHNet introduced the improved Inception module for multiscale feature extraction and the hierarchical forecast structure to guide the update of the parameters of the middle layer in the network, which enlarged the receptive field, improved the ability to control the details and global information in the image, and can predict the deformation field in real-time for unseen image pairs. MHNet performed registration evaluation on 3D brain MR scans on the publicly available dataset and compared the final registration results with traditional algorithm and deep learning-based registration models. The results showed that our method can achieve excellent registration performance. The main achievements of this work are summarized as follows:

1. MHNet is a fast unsupervised deformable registration network, which will not face the dilemma of lack of ground truth, and can register a pair of 3D MRIs within 1 s, meeting the needs of clinical medical research
2. This paper innovatively added a multiscale feature extraction module and a hierarchical forecast structure to the encoder-decoder structure to facilitate network learning and achieved better registration results than other deep learning networks
3. This paper proposed a dataset augmentation method, which can effectively expand the training data and increase the diversity of features learned by the network, thereby improving the registration performance of the model

The rest of this paper is organized as follows.  Section 2 presents the materials and our methods, including the dataset and augmentation method, the overall process of registration, network design, evaluation method, and implementation details.  Section 3 presents experimental results.  Section 4 discusses the findings based on the results, and Section 5 concludes the paper.

## 2. Materials and Methods

### 2.1. Experimental Data

This study performed registration tasks on the LONI Probabilistic Brain Atlas (LPBA40) dataset [18]. The LPBA40 dataset is public and available on the web. The data in LPBA40 was derived from *T*1-weighted brain MR scans of 40 healthy, normal volunteers, with 56 structures labeled by experts, and all image volumes had been strictly aligned with the MNI305 brain atlas. All images have original size 181 × 217 × 181 and resolution 1mm × 1mm × 1mm. We used advanced normalization tools (ANTs) [19] to perform initial affine alignment on all images. Meanwhile, all images were uniformly clipped to 160 × 192 × 160, and image intensity normalization was carried out to accelerate the speed of network convergence. We chose 1 image as the reference image, 25 images as training samples, and the remaining 14 images as test samples. Each input to the network consisted of the reference image and a training or test sample (moving image).

However, 25 training data is too sparse for CNN, the network cannot be fully trained and may even overfit. This paper proposed a dataset augmentation method. We registered the images in the training set with each other and used the obtained deformed images as new training data to expand the number of training data. This approach is mainly based on two considerations. On the one hand, all existing data registration algorithms cannot achieve 100% accuracy, and the new image generated is an intermediate image between the reference image and the moving image, which cannot completely match the reference image and the moving image. On the other hand, deep learning models, unlike traditional registration algorithms, do not iteratively learn features and calculate the deformation field required for warp, so this intermediate deformation result is nonrepetitive and efficient training data for neural networks to learn. The specific implementation method is to use the antsRegistrationSyNQuick command in ANTs to quickly register the training data, and the time to register a pair of training image volumes is only about 10s (under 8 threads). For a training dataset with the number of *N*, two original images *X* and *Y* are randomly selected. If *X* is used as the reference image and the *Y* is used as the moving image, a new training image *Y*′ can be generated by registering the two images. On the contrary, taking *Y* as the reference image and *X* as the moving image, a new deformed image *X*′ can also be generated through registration. Therefore, the number of new images *M* generated by this method can be calculated by the following equation.

(1) $$\begin{array}{c} M={\text{A}}_{N}^{2}=N\times \left(N-1\right). \end{array}$$

In this way, the dataset can be enlarged by *N* − 1 times, and the total number of training images is *N*^2^. After augmentation, the number of training images in the research had been successfully increased from 25 to 625.  Figure 1 shows the augmentation effect of our dataset in this way.

### 2.2. Registration Method

For a given pair of reference image *F* and moving image *M* defined in the 3 − *D* space domain*Ω* ⊂ *R*^3^, 3D image registration is to warp *M* through the spatial transformation *T* (i.e., deformation field *ϕ*) between *F* and *M*, so that the warped image *M*∘*ϕ* and *F* reach the optimal alignment. How to find the parameterized optimal spatial coordinate transformation through CNN was the key point of this work.  Figure 2 shows the complete architecture of the proposed registration model. This model takes the reference image *F* and the moving image *M* as input and generates a displacement vector field (DVF) after the prediction of the CNN *f*:

(2) $$\begin{array}{c} \phi =f_{\theta }\left(F,M\right), \end{array}$$

where *θ* represents the parameters of the network. Then, the STN [11] was applied to nonlinearly warp the moving image *M* with the deformation field *ϕ* (or DVF) and generate the deformed image *M*∘*ϕ*. The voxel location *i* in the moving image *M* may deviate from an integer location after being superimposed with the voxel displacement *u*(*i*) in the deformation field. But the intensities are only defined at integer locations, so the intensity of each voxel location *M*∘*ϕ*(*i*) needs to be obtained by trilinear interpolation:

(3) $$\begin{array}{c} M\circ \phi \left(i\right)=M\left(i+u\left(i\right)\right), \end{array}$$

(4) $$\begin{array}{c} M\circ \phi \left(i\right)=\underset{j\in Z\left(i^{\prime }\right)}{\sum }M\left(j\right)\underset{d\in \left\{x,y,z\right\}}{\prod }\left(1-\left|j_{d}-i_{d}^{\prime }\right|\right), \end{array}$$

where *i*′ = *i* + *u*(*i*), *𝒵*(*i*′) denotes the neighboring voxel location of *i*′, and *d* denotes the three directions in 3D space.

During the training process, the parameters of CNN *θ* are continuously updated and optimized according to the predefined loss function *L*. When there is a set of parameters that make the value of the loss function tend to the minimum (convergence), the optimal parameters $\hat{\theta }$ is obtained, which can be expressed by the following equation:

(5) $$\begin{array}{c} \hat{\theta }=\underset{\theta }{\text{argmin}}L\left(T_{\phi };F,M\right). \end{array}$$

In this registration model, the *L* consists of two parts: (1)*L*_sim_—a measure of appearance intensity difference between *F* and *M*∘*ϕ*. (2) *L*_smooth_—a regularization term that constrains the smoothing of the deformation field.

In this paper, we adopted normalized cross-correlation (NCC) [4] as the similarity measure, and its value is in [0,1]. The closer it is to 1, the higher the similarity between the two images. When used as a loss, we took its negative value, which can be expressed as the following equation:

(6) $$\begin{array}{c} L_{\text{sim}}\left(F,M,\phi \right)=-NCC\left(F,M\circ \phi \right). \end{array}$$

The deformation field predicted by CNN should be a smooth mapping to the image, but in the training process, in order to maximize the similarity between images, the deformation field is often folded and discontinuous, which is impossible in anatomy. When training is completely unsupervised, applying a spatial regularization to the generated deformation field is necessary. In addition, this move can prevent the overfitting of CNN and improve the generalization ability of the network. In this paper, the smoothness loss was penalized by introducing a spatial gradient diffusion regularization of the deformation field displacement [15]:

(7) $$\begin{array}{c} L_{\text{smooth}}\left(\phi \right)=\underset{x\in \Omega }{\sum }{\left\|\nabla u\left(x\right)\right\|}^{2}, \end{array}$$

where *u*(*x*) represents the displacement of each voxel *x* in the deformation field and *ϕ* can be parameterized by *u*(*x*). Therefore, the total loss function can be expressed as

(8) $$\begin{array}{c} L_{\text{total}}=\alpha L_{\text{sim}}\left(F,M,\phi \right)+\lambda L_{\text{smooth}}\left(\phi \right), \end{array}$$

where *α* and *λ* are trade-off parameters used to adjust the degree of similarity and regularization.

### 2.3. Multiscale Hierarchical Deformable Registration Network

MHNet adopts an encoder-decoder network structure, introducing upsampling and downsampling operations into a fully convolutional neural network to predict the DVF required for moving image warping. This structure can expand the receptive field of the network, showing strong ability in pixel-level learning. Details about MHNet are shown in Figure 3.

As the input of the network, the images *F* and *M* are concatenated in the channel dimension to form an image volume with a channel number of 2, which is passed to the network. The encoding process is similar to the calculation process of feature extraction in the classical convolutional neural network, which repeatedly applies a 3D convolutional layer with a commonly used and efficient convolution kernel of 3 × 3 × 3 and a stride of 2. The use of strided convolution can perform downsampling while extracting features, which enlarges the receptive field by halving the size of the feature maps. To extract more abstract features without changing the size of the feature map, a convolutional layer with stride 1 is added after the strided convolution. In addition, a LeakyReLu activation is designed after each convolution operation to enhance the nonlinear representation of features. After four downsamplings, the size of the feature map is only 1/16 of the input image. In the decoding stage, the size of the feature map is recovered by performing four repeated alternating operations, each of which includes, upsampling, skip connection, and convolution. The upsampling layer applies trilinear interpolation with a sampling factor of 2 to incrementally increase the feature map size. After four upsampling, the feature map is restored to the original image size, which ensures that the size of the final output DVF can be consistent with that of input images. The skip connection is to concatenate the upsampled deep feature map in the decoding path and the shallow feature map of the same size in the encoding path along the channel dimension. The combination of abstract features and concrete features enables the network to more comprehensively learn the detailed and global information in the image.

Although the encoder-decoder structure can expand the receptive field of the network to a certain extent, there are still some problems: first, the receptive fields of the first several layers in the network are still restricted by the size of the convolution kernel, while the global context information can only be reflected in the deep features. Second, existing studies have shown that with the deepening of the convolution layer, the influence from distant voxels will rapidly decay [20]. In order to avoid the suboptimal registration effect caused by insufficient receptive field size, inspired by GoogLeNet [21], this work decided to add an improved Inception module, as shown in Figure 4. In order to achieve the purpose of expanding the receptive field by increasing the size of convolution kernel, on the one hand, it is necessary to use a larger size convolution than the conventional 3 × 3 × 3. On the other hand, compared with 2D convolution, 3D convolution has a larger increase in parameters and computation. If the convolution kernel is too large, the computation will increase dramatically. At the same time, to maintain symmetry on both sides of the image in the padding operation, and to ensure that the anchor point of the convolution kernel is in the center to avoid the offset of the position information, the size of the convolution kernel mostly adopts an odd value. Therefore, the convolution kernels of 5 × 5 × 5 and 7 × 7 × 7 are suitable. Filters with convolution kernels 1 × 1 × 1, 3 × 3 × 3, 5 × 5 × 5, and 7 × 7 × 7 are used in this module. The stacking of filters of different scales enables the network to perceive image local areas of different sizes in the same layer and fuse features of different scales, so the network can output feature maps containing more spatial information. Since the use of 3D convolution will lead to a surge in the number of parameters, the bottleneck layer with a convolution kernel size of 1 × 1 × 1 is added before the large-scale filter for channel dimension reduction, so as to reduce the computational burden brought by module insertion. For a 3D convolution layer *k*, its parameter quantity *P*_*k*_ can be calculated by multiplying the number of input channels *C*_in_^*k*^ the number of output channels *C*_out_^*k*^ and the size of the convolution kernel [*H*_*k*_ × *W*_*k*_ × *D*_*k*_]:

(9) $$\begin{array}{c} P_{k}=C_{\text{in}}^{k}\times H_{k}\times W_{k}\times D_{k}\times C_{\text{out}}^{k}. \end{array}$$

By adding a bottleneck layer to reduce the dimension of the *C*_in_^*k*^, the number of input channels becomes *C*_in_^*k*^′(*C*_in_^*k*^′ < *C*_in_^*k*^). The parameter quantity of the convolution layer at this time is

(10) $$\begin{array}{c} P_{k}^{\prime }=C_{\text{in}}^{k}\times 1\times 1\times 1\times {C_{\text{in}}^{k}}^{\prime }+{C_{\text{in}}^{k}}^{\prime }\times H_{k}\times W_{k}\times D_{k}\times C_{\text{out}}^{k}. \end{array}$$

In this paper, *C*_in_^*k*^ = 2, *C*_in_^*k*^′ = 1, *C*_out_^*k*^ = 4, *H*_*k*_ = *W*_*k*_ = *D*_*k*_ ∈ {1, 3, 5, 7}. After calculation, the parameter quantity of the Inception module without adding the bottleneck layer is 3968, and the parameter quantity after adding the bottleneck layer is 1994. It can be seen that the addition of the bottleneck layer can effectively reduce the consumption of memory.

Most registration networks only rely on the deformation field generated by the end to guide the network parameter update, thus ignoring the influence of the network middle layers on the deformation field. During the training process, when the loss is responded and the gradient is back-propagated, the parameter optimization efficiency of the front-end convolution layers is far less than that of the output part at the end of the network. This situation tends to lead to insufficient network learning, slow convergence, and adverse overfitting. In order to improve this network defect, we add a hierarchical forecast structure to the network, which uses the characteristics of feature maps with different resolutions at different levels in the decoding path to predict deformation fields. Because of different levels and scales, feature maps contain different semantic information and spatial information. If the information can be fully utilized, the final deformation result will be more delicate and accurate. To realize the fusion of this information in the same dimension, the feature maps need to be upsampled with factors of 8, 4, and 2, respectively, and then three different deformation fields are obtained after convolution. The deformation fields generated by these intermediate layers can be expressed as *ϕ*_low_, *ϕ*_mid_, and *ϕ*_high_, respectively. Finally, they are concatenated with the deformation field generated at the end of the network in the channel dimension, and the deformation field with multilevel and multiscale information can be obtained after a channel dimension reduction operation. With the addition of this structure, the gradient can rapidly be propagated along the hierarchical forecast blocks, and the parameters of the intermediate layers enable to have a greater and more effective update.

### 2.4. Evaluation Method

We use visual observation to qualitatively judge the quality of the registration results and use Dice score [22] to calculate the volume overlap degree of the same anatomical tissues *S*_*f*_ and *S*_*w*_ in the reference image and the deformed image to quantitatively evaluate the registration results:

(11) $$\begin{array}{c} \text{Dice}\left(S_{f},S_{w}\right)=2\frac{\left|S_{f}\cap S_{w}\right|}{\left|S_{f}\right|+\left|S_{w}\right|}. \end{array}$$

The Dice score is between 0 and 1, with 1 representing the complete overlap of corresponding tissues in the two images. Therefore, the closer the Dice score is to 1, the better the registration effect is.

In order to verify the effectiveness of our proposed network, four advanced deformable registration algorithms were selected as baselines. The first is symmetric normalization (SyN) [23], one of the most superior traditional registration algorithms. We completed the SyN with cross-correlation as the similarity measure and gradient step size = 0.15 by using the ANTs software package. MIDIR [24] was selected as the second baseline, which is also based on unsupervised deep learning and can produce diffeomorphic deformation. In this model, the control point spacing of B-spline transformation was set as 2. In addition, we also selected the famous VoxelMorph as the baseline, which has two variants, VoxelMorph-1 and VoxelMorph-2. The loss function settings of MIDIR and VoxelMorph were the same as those in this paper, and the hyperparameters *α* and *λ* in Equation (8) were both 1. These settings had been proved to be optimal in the original text. In order to show the performance of MHNet more directly and intuitively, we also added affine transformation for comparison.

### 2.5. Implementation

MHNet was implemented using PyTorch. During the training process, considering that the memory consumption required for processing 3D images is large, we set the training batch size = 1 to avoid being out of memory. By setting different values for training, the hyperparameter values of the loss function to achieve the highest registration accuracy were determined as *α* = 1 and *λ* = 3. The model was trained for 70 epochs (43750 iterations) using ADAM gradient optimizer to ensure that the loss no longer changes significantly and the network is fully converged. The initial learning rate was set to 10-4, and after 40 epochs, the learning rate was halved to avoid the step size being too large and thus crossing the global optimal solution and falling into the local optimal solution. All experiments were performed on a single NVIDIA Tesla P100 GPU and Intel Xeon Silver 4210 CPU.

## 3. Results

### 3.1. Comparative Experimental Result

Table 1 shows the test results of MHNet and other baselines on the LPBA40 test dataset. Avg. Dice is the average Dice score calculated on all 56 anatomical structures of all test samples. At present, SyN has only found a CPU implementation. To register a pair of images in a single-threaded case, the average running time is 3914 s. To save time, this paper conducted experiments under 8 threads. It can be seen that MHNet achieves the best results in methods based on deep learning and achieves comparable performance to the state-of-the-art traditional method.  Figure 5 shows the cross-sectional results of a test sample deformed by several algorithms.

To quantitatively display the registration results in local brain regions, we selected 12 brain anatomical structures of interest.  Table 2 shows the names of these ROIs and the numbers assigned to them in this paper (we averaged the Dice score of the same structure in the left and right hemispheres into a score, such as left putamen and right putamen) and showed their average Dice score in the form of histogram in Figure 6. The results show that MHNet exhibits high registration accuracy whether based on the overall brain structure or based on the ROIs.

### 3.2. Ablation Result

This section aims to verify the impact of the improved Inception module and the hierarchical forecast structure on registration performance. Our three network variants and their registration performance were listed in Table 3. In the variant “MHNet1 (w/o Incep),” we removed the improved inception module and replaced it with a normal 3D convolution in the same place, keeping the number of input feature maps and the number of output feature maps unchanged. In MHNet2, we removed the multiscale hierarchical forecast structure. “w/o Incep+HF” is a variant that removes the improved inception module and the hierarchical prediction structure altogether, that is, leaving only the basic encoder-decoder network structure. Quantitative metrics show that the addition of these components to our network substantially improves registration accuracy.

### 3.3. Efficacy of Dataset Augmentation

The magnitude and diversity of the training data have a direct impact on the training effect of the neural network. In order to confirm whether the dataset augmentation method proposed in this paper can generate real and effective training data and have a positive impact on the performance of the proposed network, we conducted the following experiment. We trained MHNet directly on the unexpanded dataset and performed registration evaluations on the same test images. The baselines also conducted the same experiment. The experimental results (see Table 4) show that the dataset augmentation method proposed in this paper is effective in improving registration performance. MHNet learned more features and spatial information from the intermediate images between the reference images and the moving images, which improved its prediction ability. At the same time, the experimental data of baselines also shows that the approach has universal applicability, not only limited to MHNet.

## 4. Discussion

Registration based on human brain images can accurately map important brain structural regions from the brain atlas to patients' brain images during surgery, which is crucial for assisting doctors in rational surgical planning. In this study, we proposed an unsupervised deep learning registration network for brain MRI, which integrated a multiscale feature extraction module and hierarchical prediction strategy to find the optimal dense registration field, and evaluated it on the published LPBA40 dataset. The quality of the registration algorithm is generally evaluated from two aspects: accuracy and time consumption. In terms of accuracy, looking at the data in Table 1, we can see that compared with the other four existing registration methods, the method proposed in this paper exhibits the highest registration accuracy, which indicates that the proposed network has an excellent performance in aligning brain MR images. Because of the addition of the multiscale feature extraction Inception module, MHNet has a stronger ability to perceive the local area. From Figure 5, it is not difficult to see that although SyN also has a good registration performance, the deformed image generated by SyN is mostly a large global transformation in the local area. While the human cerebral cortex has many wrinkles and sulcus, so their registration needs more fine deformation. VoxelMorph uses single small-scale convolution kernels, which can make fine small deformations in local areas, but at the same time lacks the overall learning ability of local areas. However, MHNet has both of these capabilities. Other deep learning models rely only on convolution layers at the end of the network to predict the deformation field. The feature maps learned by the end convolutional layers contain deep abstract features extracted from images, but such features are prone to missing some spatial location information. They lack the design of similar hierarchical forecast structure, which makes their registration accuracy suffer constraints when deforming complex areas. In addition, during the training of the network, the gradient is back-propagated layer by layer, and the addition of the hierarchical forecast structure provides an expressway for propagation, which is conducive to the update of parameters. At the same time, through the observation of the gridded deformation field, we can realize that the deformation field predicted by MHNet has folding at the local voxel (white marked areas). Although MHNet has a higher improvement than MIDIR in registration accuracy and speed, the deformation field obtained by MIDIR is a diffeomorphic mapping with inverse consistency, which is lacking in MHNet. Therefore, our next work needs to pay more attention to the study of regularization and adopt stricter smoothing constraints on the model.

Under the same equipment, we have listed the time consumption of the algorithms mentioned in this paper in Table 1. When the registration accuracy gap is small, time consumption is the biggest advantage of MHNet over SyN. When using the SyN algorithm for registration experiments, step size needs to be manually adjusted several times to find the optimal value. However, MHNet can almost meet the needs of real-time registration and eliminates the process of manual parameter adjustment, which is very important for clinical medical research with high timeliness requirements. The time consumption of VoxelMorph is slightly less than that of MHNet, but this is negligible. At this time, the registration accuracy can better reflect the advantage of the method. Although MHNet is currently only used for brain MRI registration, it has the potential to register other organ and modal images.

## 5. Conclusions

This study presented an unsupervised learning-based full convolutional neural network for deformable image registration, called MHNet, which can quickly predict the deformation field without prior knowledge. By adding an improved Inception module and hierarchical prediction structure to the network, the problems of the narrow receptive field, the inability to update network parameters in a timely and effective manner during training, and slow convergence can be solved to a certain extent. We also used dataset augmentation to improve the performance of MHNet again. By comparing with other traditional or deep learning-based methods, MHNet has been proven to have superior performance in terms of registration accuracy and time consumption.

## Figures and Tables

**Figure 1:** Cross-sectional slices of images at the same location. (a, b) The original training images. (c, d) The augmented new images.

**Figure 2:** The overall framework of the proposed registration model. The solid and dashed lines represent the process of feedforward calculation and gradient backpropagation, respectively.

**Figure 3:** Architecture of the multiscale hierarchical deformable registration network.

**Figure 4:** Schematic diagram of inception multiscale feature extraction module.

**Figure 5:** Visualization results of several registration methods employed in this paper. The first row shows, from left to right, the reference image, moving image, and the meshed deformation field and deformed image produced by the MHNet. The second row shows the deformed images of the moving image warped by SyN, MIDIR, VoxelMorph-1, and VoxelMorph-2.

**Figure 6:** Histogram of Dice scores for anatomical structures of interest for SyN, MIDIR, VoxelMorph-1, VoxelMorph-2, and MHNet.

**Table 1:** Average Dice scores of Affine, SyN, VoxelMorph-1, VoxelMorph-2, MIDIR, and MHNet.

Method	Avg. Dice	Time (s)
Affine	0.642 ± 0.017	
SyN	0.706 ± 0.013	782 (CPU)
MIDIR	0.680 ± 0.010	1.06 (GPU)
VoxelMorph-1	0.699 ± 0.011	0.08 (GPU)
VoxelMorph-2	0.704 ± 0.011	0.24 (GPU)
MHNet	0.707 ± 0.010	0.29 (GPU)

**Table 2:** Names of brain ROIs selected in the LONI LPBA40 dataset.

Number	Name	Number	Name
1	Insular cortex	7	Middle temporal gyrus
2	Lingual gyrus caudate	8	Angular gyrus
3	Putamen	9	Middle occipital gyrus
4	Hippocampus	10	Gyrus rectus
5	Inferior frontal gyrus	11	Cerebellum
6	Superior parietal gyrus	12	Brainstem

**Table 3:** Results of MHNet ablation studies.

Variant	Avg. Dice	Time (s)
MHNet1 (w/o Incep)	0.703 ± 0.012	0.22 ± 0.06
MHNet2 (w/o HF)	0.704 ± 0.011	0.26 ± 0.06
MHNet3 (w/o Incep+HF)	0.701 ± 0.012	0.19 ± 0.06
MHNet	0.707 ± 0.010	0.29 ± 0.07

**Table 4:** Dice scores on the original and augmented datasets of MIDIR, VoxelMorph-1, VoxelMorph-2, and MHNet.

Model	Avg. Dice (original)	Avg. Dice (augmented)
MIDIR	0.671 ± 0.013	0.680 ± 0.010
VM-1	0.690 ± 0.013	0.698 ± 0.011
VM-2	0.697 ± 0.012	0.703 ± 0.013
MHNet	0.698 ± 0.010	0.707 ± 0.010

## Data Availability

The data supporting this study are from previously reported studies and dataset, which have been cited. The processed data are available from the corresponding author upon request.
